RETRACTED

# Association of Lower Extremity Vascular Disease, Coronary Artery, and Carotid Artery Atherosclerosis in Patients with Type 2 Diabetes Mellitus

**DOI:** 10.1155/2021/6268856

**Published:** 2021-10-16

**Authors:** Zheng Yang, Bing Han, Hongguang Zhang, Guohui Ji, Liang Zhang, Bhupesh Kumar Singh

**Affiliations:** ^1^Vascular Surgery, No. 2 Hospital of Baoding, Baoding 071000, China; ^2^Arba Minch Institute of Technology, Arba Minch University, Ethiopia

## Abstract

The motive of this article is to present the case study of patients to investigate the association between the ultrasonographic findings of lower extremity vascular disease (LEAD) and plaque formation. Secondly, to examine the association between the formation of coronary artery and carotid artery atherosclerosis in patients with type 2 diabetes mellitus. 124 patients with type 2 diabetes (64 males and 60 females with the age group 25-78 years) are considered for the research studies who have registered themselves in the Department of Endocrinology and Metabolism from April 2017 to February 2019. All participants have reported their clinical information regarding diabetes, alcohol consumption, smoking status, and medication. The blood samples from subjects are collected for measurement of HbA_1c_, total cholesterol, triglycerides, HDL-c, and LDL-c levels. Two-dimensional ultrasound has been used to measure the inner diameter, peak flow velocity, blood flow, and spectral width of the femoral artery, pop artery, anterior iliac artery, posterior tibial artery, and dorsal artery and to calculate the artery stenosis degree. Independent factors of atherosclerosis are determined by multivariate logistic regression analysis. The results are evaluated within the control group and it is found that there is no significant impact of gender, age, and body mass index (*P* > 0.05) on the lower extremity vascular diseases. Those with smoking, alcohol consumption, hypertension, and dyslipidemia have higher positive rate (*P* < 0.05). The type 2 diabetes mellitus group has higher diastolic blood pressure and lower triglyceride (*P* < 0.05). Diastolic blood pressure, HbA_1C_, total cholesterol, HDL-c, and LDL-C are not remarkably dissimilar between the type 2 diabetes mellitus group and the control group (*P* > 0.05). Compared with the control group, the type 2 diabetes mellitus group has higher frequency of lower extremity vascular diseases in the dorsal artery than in the pop artery (*P* < 0.05). The blood flow of type 2 diabetes mellitus group is found to be lower than that of the control group, especially in the dorsal artery (*P* < 0.05). The blood flow velocity of the dorsal artery is accelerated (*P* < 0.01). Among 117 patients of type 2 diabetes mellitus (94.35%) with a certain degree of injury, there are 72 cases of type I carotid stenosis (58.06%), 30 cases of type II carotid stenosis (24.19%), and 15 cases of type III carotid stenosis (12.10%). Out of 108 subjects in the control group, there are 84 cases of type 0 carotid stenosis (77.78%), 19 cases of type I carotid stenosis (17.59%), 5 cases of type II carotid stenosis (4.63%), and 0 case of type III carotid stenosis (0.00%). Compared with the control group, carotid stenosis is more common in patients with type 2 diabetes mellitus (*P* < 0.05). Age, smoking, duration of diseases, systolic blood pressure, and degree of carotid stenosis are found to be associated with atherosclerosis. The findings suggest that the color Doppler ultrasonography can give early warning when applied in patients with carotid and lower extremity vascular diseases to delay the incidence of diabetic macroangiopathy and to control the development of cerebral infarction, thus providing an important basis for clinical diagnosis and treatment.

RETRACTED

## 1. Introduction

Lower extremity vascular disease (LEAD) is the main manifestation of peripheral artery disease. It represents systemic atherosclerosis involving peripheral blood vessels, thus is related to the increased risk of cardiovascular diseases (CVD) [1]. Lower extremity vascular diseases in patients with diabetes mellitus generally cannot be detected clinically in the early stages due to the common complications of neuropathy [2, 3]. Patients with diabetes mellitus usually are unaware of the fact that the early progress of lower extremity vascular disease is due to the loss of pain and the decreasing frequency of intermittent claudication, until the symptoms get worsen and the disease turns into an ulcer or gangrene, which usually occurs at the last stage of the lower extremity vascular disease and eventually leads to amputation [4, 5]. Therefore, the early diagnosis and treatment of diabetes patients requires the index of early lower extremity vascular disease, which helps in avoiding amputation and in improving the living quality of patients [6, 7]. Color Doppler ultrasonography is a simple, convenient and feasible noninvasive technology, which can accurately locate and observe the characteristics of vascular diseases and the formation of lower limb plaques in patients with diabetes mellitus [8]. At the same time, it can detect and distinguish the formation of carotid atherosclerotic plaque and find out the potential risk factors of patients with diabetes mellitus to provide basis for early clinical diagnosis, treatment, rehabilitation, and intervention [9–11]. Therefore, the purpose of this study is to discuss the association between ultrasonic manifestations of lower extremity vascular disease and plaque formation, plus the association between the coronary artery and carotid artery atherosclerosis in patients with type 2 diabetes mellitus, so as to guide the clinical diagnosis and treatment.

RETRACTED

### 1.1. Literature Review

There are many research studies which revolves around the area of research discussed in this paper, and a few recent studies have been discussed in this subsection.

In [12], the authors claim that LEAD needs a strict monitoring of CVD risk factors such as diabetes, blood pressure, and age. The correlation between the glucose control and LEAD is not identified till date. The authors have tried to find out the correlation between LEAD and glucose levels in the patients to minimize the risk of CVDs. The authors have suggested that more factors are to be studied to establish the relationship between diabetes and LEAD in diabetic patients. In [13], the authors have analyzed data for atherosclerosis, where blood pressure extremities are evaluated in around 6000 Americans between the age group of 45 to 84. The artery disease is found in 23% of patients out of 1000 patients whose ankle-brachial index is less than 0.9. The article [14] provides a comprehensive overview of the epidemiology of peripheral artery ailments in diabetic patients. An analysis is also presented about the metabolism issues in diabetic patients that cause plaque instability in the diabetic patients. The study outcome shows that diabetic patients are prone to artery ailments, ulcers, and limb ischemia.

In [15], authors have performed analysis on genes related to type 2 (T2) diabetes mellitus. They have analyzed risk factors related to genes for diabetic patients. T2 diabetic patients have shown remarkable changes in differentially exposed genes. Among these, VEGFA gene is correlated with several healthcare complications in T2 diabetic patients. A few genes cause obesity, inflammation, and stress in T2 diabetic patients. In [16], it is explained that patients shows poorer prognosis for damaged limbs if they are suffering from diabetes as compared to nondiabetic patients. A regular screening for LEAD in patients of T2 diabetes mellitus is suggested. This article presents current evidences about LEAD in diabetic patients in order to explore the management options for LEAD in diabetic patients. In [17], the authors have identified the association of physical activities with diabetes mellitus. The impact of hypertension is also studied with diabetes mellitus. The study group is classified into four categories, no activity, minimal activity, insufficient activity, and regular activity in diabetic patients, and then, the health issues are observed of diabetic patients. It is found that regular activity improves health concerns in diabetic patients even they are related to LEAD. In [18], the authors have taken up study on exhaled breath for diagnosis of lethal diseases including diabetes and cardiovascular diseases. The impact of toxic contents in the exhaled breath can be used to diagnose various serious ailments in the human body. In [19], the authors have studied LOX-1 as a biomarker for identification of LEAD disease in T2 diabetic patients.

RETRACTED

In [20], authors have studied the signs of atherosclerosis in patients of T2 diabetes, and it is found that T2 diabetic patients are at increased risk. In [21], a study is presented of LADA patients with T2 diabetes and T1 diabetes. Initially, no patient has registered with CVD history. All patients were scanned to catch atheroma plaques. The plaque is found in diabetic patients, and it is concluded that diabetic patients can develop heart risks at any stage of diabetes. In [22], the subjects are 523 patients with T2 diabetes mellitus, and the study is conducted to estimate 10-year risk of CVDs. In the study, serum cystatin C level is found to be associated with atherosclerosis. This outcome suggests that high cystatin C level can be used as biomarker for measuring the risk of CVD in patients with T2 diabetes mellitus. In [23], the authors have studied association of kidney disease and atherosclerotic in T2 diabetic patients. The kidney disease is first to occur in T2 diabetic patients, and this kidney disease can become a major cause of cardiovascular diseases in T2 diabetic patients. In [24], the authors have made assessment of inflammation biomarkers for atherosclerosis in T1 diabetes mellitus. In [25], a relationship is studied between carotid atherosclerosis and T2 diabetic patients.

There are many studies as mentioned above and mentioned in [26, 27] which reveal the association of diabetic patients and vascular diseases.

This paper is conducting a research study for proving the same. The major findings of the paper are given below.

- The subjects are 124 patients with type 2 diabetes mellitus (64 males and 60 females, aged from 25 years old to 78 years old) and are considered for case study
- Fasting blood samples were collected from each subject after fasting for 10 hours to measure the levels of glycated hemoglobin A_1c_ and HbA1c, total cholesterol, triglyceride, high-density lipoprotein cholesterol (HDL-c), and low-density lipoprotein cholesterol (LDL-c)
- The diagnosis of diabetes mellitus is based on the 2010 standards of American Diabetes Association. Atherosclerotic plaque is defined as the focal structure invading the arterial cavity with a size of at least 0.5 mm or at least 50% greater than the thickness of the surrounding vessel wall
- Compared with the control group, the incidence of lower extremity vascular diseases in dorsal artery was higher than that in pop artery in type 2 diabetes mellitus group
- The findings are stated with statistical parameters in results section

The paper is arranged into 5 parts. First part begins with introduction, and then, literature review is covered. The major findings are also mentioned in this part. The next part describes data and methods. The third part explains results of the paper. The last part concludes the case study of T2 diabetic patients for vascular diseases.

RETRACTED

## 2. Data and Methods

### 2.1. Selection Criteria and Assumptions

*Subject information:* 124 patients with type 2 diabetes mellitus are selected as subjects of the case study (64 males and 60 females, aged from 25 years old to 78 years old) who were hospitalized in the Department of Endocrinology and Metabolism of No. 2 Hospital of Baoding, China, from April 2017 to February 2019.

*Inclusion criteria:* Gender was not given importance; patients of all genders diagnosed with type 2 diabetes mellitus over 18 years of age were considered as subjects.

*Exclusion criteria:* Patients with type 1 diabetes mellitus; patients with gestational diabetes mellitus; patients with other specific types of diabetes mellitus; patients with hepatic insufficiency (acute severe hepatitis; alanine aminotransferase, or aspartate aminotransferase > 1.5 times the upper limit of normal) and renal insufficiency (serum creatinine ≥ 115 *μ*mol/L, or glomerular filtration rate < 60 mL/min/1.73 m^2^); patients with hypothyroidism; patients with acute infection; patients with malignant tumors; patients with mental illness.

*Medical ethics:* This study was approved by the Ethics Committee of the Hospital. All participants had signed informed consent before registration.

### 2.2. Methods

#### 2.2.1. Laboratory Measurement

Fasting blood samples were collected from each subject after fasting for 10 hours to measure the levels of glycated hemoglobin A_1c_ and HbA1c, total cholesterol, triglyceride, high-density lipoprotein cholesterol (HDL-c), and low-density lipoprotein cholesterol (LDL-c).

#### 2.2.2. Ultrasonography

Acuson Sequoia 512 scanner equipped with 5-13 MHz linear array transducer was used for color Doppler ultrasonography of lower limb artery in all patients. During the examination, the angle between ultrasonic beam and blood flow was less than 60°. Two-dimensional ultrasound was used to visually detect the condition of vessel wall, intima, and cavity along anatomical position via femoral artery, pop artery, anterior tibial artery, posterior tibial artery, and dorsal artery, and then, observation was done for the intravascular blood flow and cavity and color Doppler blood flow imaging. Sampling of blood vessels with pulse width was carried out to obtain the maximum blood flow spectrum. The shape of the spectrum was also examined to determine the inner diameter, peak flow velocity, blood flow, and spectral width. The artery stenosis degree was calculated by the following formula: stenosis degree = (vascular inner diameter − effective diameter of blood vessel)/vascular inner diameter × 100%.

RETRACTED

The classification of stenosis is as follows: type 0: no stenosis; type I: stenosis accounts for 1% to 19%; type II: stenosis accounts for 20% to 49%; type III: stenosis accounts for 50% to 99%. The last step was to observe whether there are plaques in carotid artery and lower limb artery.

#### 2.2.3. Diagnostic Criteria

The diagnosis of diabetes mellitus is based on the 2010 standards of American Diabetes Association. Atherosclerotic plaque is defined as the focal structure invading the arterial cavity with a size of at least 0.5 mm or at least 50% greater than the thickness of the surrounding vessel wall.

### 2.3. Statistical Analysis

SPSS 17.0 software package was used for statistical analysis. All variables were tested for normality. Normal distribution data and measurement data were expressed as median ± standard deviation (SD), and skew data were expressed as median within quartile. Classification variables were expressed as percentages (%).

- Comparisons of normal distribution data and skewed data between groups were conducted by unpaired Student's *t* test and Mann-Whitney *U* test, respectively. Chi-square test was used to compare classified variables between groups. Logical return analysis was carried out to determine various factors related to atherosclerosis. Odds ratio (OR) was calculated to determine whether the related factors were risk factors of atherosclerosis. Multivariate linear return analysis was performed to identify the independent related factors of atherosclerosis. *P* value < 0.05 for both tails was considered as an indication of statistically significant difference

## 3. Results

### 3.1. Clinical Characteristics of Subjects

A total of 124 eligible consenting patients participated in the study, including 64 male patients and 60 female patients, aged between 25 and 85 years, with an average age of 53.24 ± 6.16 years. Their course lasted from 1 to 35 years, with an average course of 9.6 ± 2.7 years. The control group had 55 healthy male patients and 53 female patients, aged between 27 and 81 years, with an average age of 52.28 ± 4.87 years. There were no differences in sex, age, and body mass index between two groups (*P* > 0.05), but the patients with smoking, drinking, hypertension, and dyslipidemia had higher positive rate (*P* < 0.05) as shown in Table 1.

RETRACTED

### 3.2. Clinical Data of Subjects

Compared with the control group, the type 2 diabetes mellitus group had higher diastolic blood pressure and lower triglyceride (*P* < 0.05). However, there was no significant difference in diastolic blood pressure, HbA1C, total cholesterol, HDL-c, and LDL-C between two groups (*P* > 0.05) as shown in Table 2.

### 3.3. Comparison of Hemorheological Indexes between Two Groups

Compared with the control group, the incidence of lower extremity vascular diseases in dorsal artery was higher than that in pop artery in type 2 diabetes mellitus group (*P* < 0.05). The blood flow of type 2 diabetes mellitus group was lower than that of the control group, especially in the dorsal artery (*P* < 0.05). The blood flow velocity of dorsal artery was increased (*P* < 0.01). The blood flow spectrum increased in different degrees, and the blood flow spectrum of dorsal artery was higher than that of pop artery (*P* < 0.01). Therefore, the data of our study showed that the change of dorsal artery was the most significant, and all arterial injuries were bilateral or multiple arterial diseases of lower extremity arterial disease in patients with diabetes mellitus as shown in Figure 1 and values are given in Table 3. Figure 1 depicts that T2 diabetic patients have lower flow of blood than the control group. The arterial injuries were bilateral or multiple arterial diseases; LEAD is found in patients with diabetes mellitus.

### 3.4. Comparison of Degrees of Carotid Stenosis between Two Groups

In this study, 117 patients with type 2 diabetes mellitus (94.35%) had certain degree of injury, including 72 cases of type I carotid stenosis (58.06%), 30 cases of type II carotid stenosis (24.19%), and 15 cases of type III carotid stenosis (12.10%). Among the 108 subjects in the control group, there were 84 cases of type 0 carotid stenosis (77.78%), 19 cases of type I carotid stenosis (17.59%), 5 cases of type II carotid stenosis (4.63%), and 0 case of type III carotid stenosis (0.00%). Type 2 diabetes mellitus group had more carotid stenosis cases than the control group (*P* < 0.05) as displayed in Table 4.

The ultrasound positive rate was 45.16% (56 cases) in carotid artery, 45.97% (57 cases) in the lower extremity artery, and 80.65% (100 cases) in the carotid artery + lower extremity artery (*P* < 0.05).

RETRACTED

### 3.5. Positive Rate of Atherosclerosis

The ultrasonic positive rate of carotid artery was 56 (45.16%), lower extremity artery was 57 (45.97%), and carotid artery+lower extremity artery was 100 (80.65%)(*P* < 0.05) as given in Table 5.

### 3.6. Determination of the Independent Factors of Atherosclerosis by Multivariate Logical Return Analysis

In multivariate logic analysis, gender, age, body mass index, smoking, drinking, hypertension, dyslipidemia, systolic blood pressure, diastolic blood pressure, HbA1C, total cholesterol, triglyceride, HDL-c, and LDL-C were taken as independent variables. The analysis confirmed that age, smoking, course of disease, systolic blood pressure, and carotid stenosis were associated with atherosclerosis as displayed in Figure 2 and Table 6.

### 3.7. Description on Results

Complications of atherosclerosis lead to the excessive morbidity and mortality of patients with diabetes mellitus. Therefore, early detection of atherosclerosis is extremely important for patients with type 2 diabetes mellitus to prevent various cardiovascular events, such as myocardial infarction, stroke, and death. Ultrasonic scanning is a noninvasive, accurate, and cheap technique for detecting early atherosclerotic plaque and arterial wall changes [28]. Therefore, in this study, ultrasonography is used for early detection of atherosclerosis. The main pathological changes of vascular diseases in neck and lower limbs of patients with diabetes mellitus are thickening of intima-media thickness, narrowing of vascular cavity, and decrease of compliance in walls [29]. Irregular atherosclerotic plaque leads to further narrowing of the cavity in the intima of blood vessels and then secondary thrombosis and even vascular occlusion [16]. The vascular disease of patients with diabetes mellitus is similar to that of patients without diabetes mellitus. However, the incidence of diabetes is high, and atherosclerosis progresses rapidly, which thickens the carotid intima-media and the proximal intima of internal carotid artery and even causes plaque [19].

The manifestations of diabetic lower extremity arterial disease are usually thickened arterial intima, lacking or uneven, and some atherosclerotic plaques of different sizes protrude into the cavity, resulting in different degrees of arterial stenosis or even blocking arterial stenosis [20]. When there is stenosis, the blood flow is weakened, and the spectrum is widened and filled but no normal three-phased wave is found. Where there is a blockage, the wall of blood vessels decreases, and the cavity disappear. Achromatic blood flow shows that the spectrum of blood flow is invalid, and the blood flow signal of distal stenosis is weakened. Pulse Doppler shows that the peak systolic velocity is low. This study found that patients with type 2 diabetes have more carotid stenosis cases than the control group. Compared with the control group, the incidence of lower extremity vascular diseases of dorsal artery was higher than that of pop artery in type 2 diabetes mellitus group. Blood flow in type 2 diabetes mellitus group was lower than that in control group, especially in dorsal artery.

RETRACTED

Blood flow spectrum increased in different degrees, and the blood flow spectrum of dorsal artery was higher than that of pop artery. Therefore, the data of our study depicted that the change of dorsal artery was the most significant, and all arterial injuries were bilateral or multiple arterial diseases of lower extremity arterial disease in patients with diabetes mellitus. We assessed the prevalence rate of atherosclerosis in hospitalized Chinese patients with type 2 diabetes mellitus. The data of our study proved that the prevalence rate of atherosclerosis in all Chinese patients diagnosed with type 2 diabetes was 80.65% (100/124 cases). However, if only based on carotid ultrasonography, the positive rate of atherosclerosis was only 45.16% (56/124 cases). According to ultrasonography of carotid artery and lower limbs, the positive rate increased to 80.65%. Some studies have shown that carotid atherosclerosis is related to atherosclerosis in other parts and can be used as an index of systemic atherosclerosis [21, 22]. Carotid atherosclerosis cannot be used to predict atherosclerosis in other parts of the arterial system. Therefore, it may have important clinical value to use the ultrasonography of carotid artery and lower limb to detect the existence of atherosclerosis. If only one of these tests is measured, the severity of atherosclerosis in patients may be underestimated.

Our results also proved that the prevalence rate of atherosclerosis in patients with type 2 diabetes mellitus increases with age and the course of diabetes mellitus. Compared with young patients, the prevalence rate of atherosclerosis in elderly patients was higher, and plaque was more likely to occur in advanced staged patients with type 2 diabetes mellitus. Similar to other studies, we found that some traditional risk factors of atherosclerosis also exist in patients with type 2 diabetes mellitus. In our study, the binary logic return model proved that atherosclerotic plaque was related to age, smoking, course of disease, systolic blood pressure, and carotid stenosis. Our data proved that patients with type 2 diabetes mellitus and atherosclerosis were more likely to suffer from complicated cardiovascular and cerebrovascular diseases than those without atherosclerosis. The incidence of cardiovascular and cerebrovascular events was significantly higher in patients with carotid artery and lower extremity atherosclerosis than that in patients with carotid artery or lower extremity atherosclerosis.

RETRACTED

To sum up, color Doppler ultrasonography has high sensitivity, convenient examination, and good repeatability, which greatly improves the positive rate of lower extremity vascular disease and has important guiding significance for early clinical diagnosis, prevention, and treatment of diabetic carotid artery and lower extremity vascular diseases. Ultrasonography could give early warning when applied in patients with carotid and lower extremity vascular disease to delay the incidence of macroangiopathy and slow the development of cerebral infarction and other macroangiopathy, thus providing an important basis for clinical diagnosis and treatment.

## 4. Conclusion

In this article, the investigation of association between LEAD and plaque formation and between carotid artery atherosclerosis and T2 diabetic patients is performed. The results are evaluated within the control group and 124 diabetic patients (type 2 diabetes). The findings suggest that T2 diabetes mellitus group has higher diastolic blood pressure (DBP) and lower triglyceride (*P* < 0.05). DBP, HbA1C, total cholesterol, HDL-c, and LDL-C are not remarkably dissimilar between the T2 diabetes mellitus group and the control group (*P* > 0.05). Compared with the control group, the T2 diabetes mellitus group has higher frequency of lower extremity vascular diseases in the dorsal artery than in the pop artery (*P* < 0.05). The blood flow of T2 diabetes mellitus group is found to be lower than that of the control group, especially in the dorsal artery (*P* < 0.05). Among 124 patients of T2 diabetes mellitus (94.35%) with a certain degree of injury, there are 72 cases of type I carotid stenosis (58.06%), 30 cases of type II carotid stenosis (24.19%), and 15 cases of type III carotid stenosis (12.10%). Out of 108 subjects in the control group, there are 84 cases of type 0 carotid stenosis (77.78%), 19 cases of type I carotid stenosis (17.59%), 5 cases of type II carotid stenosis (4.63%), and 0 case of type III carotid stenosis (0.00%). Compared with the control group, carotid stenosis is more common in patients with T2 diabetes mellitus (*P* < 0.05). The ultrasound positive rate is 45.16% (56 cases) in carotid artery, 45.97% (57 cases) in the lower extremity artery, and 80.65% (100 cases) in the carotid artery + lower extremity artery (*P* < 0.05). Age, smoking, duration of diseases, systolic blood pressure, and degree of carotid stenosis are found to be associated with atherosclerosis. It can be concluded that Color Doppler ultrasonography could give early warning when applied in patients with carotid and LEAD to delay the incidence of diabetic macroangiopathy and to control the development of cerebral infarction, thus providing an important basis for clinical diagnosis and treatment.

RETRACTED

## Figures and Tables

**Figure 1:** Comparison of hemorheological indexes.

**Figure 2:** Vascular stenosis degree age. Age was positively correlated with the degree of vascular stenosis.

**Table 1:** Clinical characteristics of subjects.

Item	Control group	Type 2 diabetes mellitus group	*χ* ^2^/*t* value	*P* value
Gender (male : female)	55 : 53	64 : 60	5.372	0.374
Age	52.28 ± 4.87	53.24 ± 6.16	1.184	0.452
Body mass index	24.18 ± 2.46	24.37 ± 2.55	1.322	0.186
Smoking (%)	16 (14.81%)	29 (23.39%)	3.675	0.031
Drinking (%)	24 (22.22%)	32 (25.81%)	5.964	0.025
Hypertension (%)	25 (23.15%)	37 (29.84%)	4.375	0.015
Dyslipidemia	28 (25.93%)	45 (36.29%)	3.216	0.013

**Table 2:** Clinical data of subjects.

Item	Control group	Type 2 diabetes mellitus group	*χ* ^2^/*t* value	*P* value
Systolic blood pressure (mmHg)	122.34 ± 13.74	135.35 ± 15.48	3.678	0.014
Diastolic blood pressure (mmHg)	79.85 ± 9.26	80.04 ± 10.13	2.547	0.472
HbA1C (%)	9.01 ± 2.13	9.34 ± 2.04	1.132	0.156
Total cholesterol (mmol/L)	4.71 ± 0.84	4.72 ± 0.96	5.964	0.347
Triglyceride (mmol/L)	2.08 ± 0.64	1.62 ± 0.37	3.257	0.024
HDL-c (mmol/L)	1.08 ± 0.27	1.13 ± 0.22	5.186	0.338
LDL-C (mmol/L)	3.05 ± 0.47	3.07 ± 0.58	1.159	0.624

**Table 3:** Comparison of hemorheological indexes between two groups.

Position	Group	Vascular inner diameter	Peak velocity	Blood flow	Spectral width
Left femoral artery	Control group	7.48 ± 1.12	0.85 ± 0.16	42.3 ± 4.88	5.23 ± 1.31
	Type 2 diabetes mellitus group	6.94 ± 0.89	0.93 ± 0.15	38.74 ± 5.53	6.14 ± 1.06
Right femoral artery	Control group	7.11 ± 0.67	0.86 ± 0.12	36.43 ± 3.54	5.82 ± 1.15
	Type 2 diabetes mellitus group	7.15 ± 0.73	0.92 ± 0.28	37.13 ± 4.24	6.73 ± 1.06
Left pop artery	Control group	5.92 ± 0.47	0.48 ± 0.13	13.82 ± 1.15	4.26 ± 0.15
	Type 2 diabetes mellitus group	5.18 ± 0.16^a^	0.72 ± 0.16^a^	14.57 ± 3.13	5.84 ± 0.28^b^
Right pop artery	Control group	5.71 ± 0.43	0.52 ± 0.16	14.28 ± 2.87	4.73 ± 0.55
	Type 2 diabetes mellitus group	5.32 ± 0.85	0.67 ± 0.16	11.38 ± 2.97	5.95 ± 1.13^a^
Dorsal artery of left foot	Control group	1.93 ± 0.22	0.35 ± 0.14	1.29 ± 0.37	4.06 ± 1.08
	Type 2 diabetes mellitus group	1.32 ± 0.29^b^	0.53 ± 0.09^a^	0.73 ± 0.15^a^	5.96 ± 1.88^b^
Dorsal artery of right foot	Control group	2.04 ± 0.87	0.35 ± 0.22	1.63 ± 0.26	4.15 ± 0.87
	Type 2 diabetes mellitus group	1.16 ± 0.23^b^	0.73 ± 0.11^a^	0.83 ± 0.26^a^	6.34 ± 2.56^b^
*t* value		5.87	6.13	3.25	4.18
*F* value		0.014	0.023	0.011	0.015

Note: ^a^ represents for *P* < 0.05 and ^b^ stands for *P* < 0.01 (comparison between two groups).

RETRACTED

**Table 4:** Degree of carotid stenosis.

Group	Type 0	Type I	Type II	Type III
Control group	84 (77.78%)	19 (17.59%)	5 (4.63%)	0 (0.00%)
Type 2 diabetes mellitus group	7 (5.65%)	72 (58.06%)	30 (24.19%)	15 (12.10%)
*χ* ^2^/*t* value	3.645	6.528	5.146	4.332
*P* value	0.011	0.08	0.013	0.006

**Table 5:** Positive rate of atherosclerosis.

Item	Positive rate
Carotid ultrasonography	56 (45.16%)
Lower extremity ultrasonography	57 (45.97%)
Carotid artery+lower extremity ultrasonography	100 (80.65%)
*χ* ^2^ value	6.437
*P* value	0.006

**Table 6:** Independent factors of atherosclerosis were determined by multivariate logical return analysis.

Item	*β*	SE	OR (95% CI)	*P* value
Age	0.148	0.015	1.237 (1.052-1.426)	<0.001
Smoking	0.234	0.024	1.264 (1.017-1.483)	0.003
Course of disease	0.016	0.064	1.058 (0.973-1.228)	0.006
Systolic blood pressure	0.058	0.037	1.022 (0.875-1.137)	0.005
Degree of carotid stenosis	0.527	0.018	2.246 (2.172-2.463)	<0.001

## Data Availability

Data will be made available on request.
